# Analyzing the Prospects of Blockchain in Healthcare Industry

**DOI:** 10.1155/2022/3727389

**Published:** 2022-12-02

**Authors:** Shilpa Srivastava, Millie Pant, Sunil Kumar Jauhar, Atulya K. Nagar

**Affiliations:** ^1^Christ (Deemed to be University), Delhi NCR, India; ^2^Indian Institute of Technology Roorkee, Roorkee, India; ^3^Indian Institute of Management, Kashipur, India; ^4^Liverpool Hope University, UK

## Abstract

Deployment of secured healthcare information is a major challenge in a web-based environment. eHealth services are subjected to same security threats as other services. The purpose of blockchain is to provide a structure and security to the organization data. Healthcare data deals with confidential information. The medical records can be well organized and empower their propagation in a secured manner through the usage of blockchain technology. The study throws light on providing security of health services through blockchain technology. The authors have analyzed the various aspects of role of blockchain in healthcare through an extensive literature review. The application of blockchain in COVID-19 has also been analyzed and discussed in the study. Further application of blockchain in Indian healthcare has been highlighted in the paper. The study provides suggestions for strengthening the healthcare system by blending machine learning, artificial intelligence, big data, and IoT with blockchain.

## 1. Introduction

The induction of IT Tools and techniques in medical domain have shown a remarkable impact and provided a wide opportunity in various ehealth services. These online services are prone to same kinds of threats as other online applications. Security is one of the pertinent issues for the effective and successful implementation of these ehealth services. Healthcare data is versatile and huge in nature which when transferred to its different stakeholders require high degree of integrity, confidentiality, and availability. The different stakeholders of healthcare services like doctors, patients, nurse, paramedical staff, official staff, etc. have different roles to play and for maintaining privacy not all the data should be shared to all the users [1]. In the recent years, blockchain has shown a remarkable impact in sharing the data in a secured manner. Different services have been highly benefited by inculcating blockchain. Its significance can be easily analyzed in health services also. The medical records and information can be easily streamlined in a protected environment. The blocks created by one user are confirmed by millions of computers leading towards a unique record with unique history, even if a single record is disrupted it disrupts the complete chain having millions of instances. In the current scenarios, many industries are looking forward to apply blockchain technology for securing their data. In the news industry, as well as in social media, it is pertinent that only the reliable news should be propagated. The detection and identification of fake news is the need of the hour. In the era of digitization, it is not difficult to manipulate and post the digital content on social media. The integration of blockchain can control the propagation of fake news. In the medical domain the maintenance and security of electronic health record has always been on high priority. It involves all the stakeholders of medical services. EHR framework can be developed through the blockchain technology which shall help in providing immutable and authentic medical records over a broader network. The risk involved in maintaining the personal health data can be minimized to a greater extent through the blockchain-based solution.

The integration with technologies like artificial technology can ensure seamless sharing of data among different stakeholders while safeguarding data privacy. Blockchain technology also empowers interorganizational services or workflows in real time, be the users, inside and outside the national health systems anywhere in the world. In case of people moving from one place to another, it is mandatory to strengthen and disseminate the migrant health information enabling analytics for strategic decisions. Blockchain technology can emerge as a strong digital tool to improve communication and overcome gaps in medical data sharing. The requirements of blockchain-based data governance model can also be analyzed for COVID-19 digital health certificates.

The study focuses on the different blockchain issues, history, its process, benefits, and different challenges for the wide deployment. This paper has 10 sections.  Section 2 describes the blockchain technology, its history, different applications, different types, and the algorithms being used. The inculcation of blockchain in healthcare especially in pandemic time (COVID-19) has been discussed in section 3.  Section 3 also discusses the status of blockchain in Indian healthcare scenario.  Section 4 throws light on the literature review based on the application of blockchain in healthcare services followed by its analysis in section 5. Different issues like challenges and disadvantages have been analyzed and described in section 6.  Section 7 mentions the difference of the study from the previous studies. Some of the pertinent recent studies have been discussed in section 8. Various suggestions have been provided in section 9, and finally, the study is concluded in section 10.

## 2. Blockchain- A Brief Overview

The invention of blockchain took place in the year 1991 by two scientists Stuart Haber and W. Scott Stornetta 17 years before the release of the Bitcoin paper by Satoshi Nakomoto's Bitcoin paper (2008). The proposed idea was to calculate hash values of documents and saving them along with a timestamp. Data structure is used for linking the records by incorporating the hashes of previous record's certificates which when applied to digital signatures makes the time stamping process sustainable [2]. Basically, it can be considered as recording, storing, and transferring records in a distributed environment in a secured fashion. The reason behind its widespread acclaim lies on the three main properties that include decentralization, transparency, and immutability. Decentralization means that there is no central authority, transactions are stored, and distributed across all the network participants which makes difficult for the hacker to corrupt. Blockchain follows peer-to-peer transactions and partitions its entire workload between all the network participants. A linked list containing data and a hash pointer pointing to the previous block is maintained and even if there is a slight change in data the hash will be changed which in turn change the hash of previous block and so on. This will completely change the chain, which is impossible. This is how blockchain attain immutability.

### 2.1. Advantages

The blockchain technology is a new concept but still it has shown its worth and importance in a very short period time. Here is a list of some key advantages of the blockchain technology [Figure 1].

### 2.2. Types of Blockchain

Primarily there are two types of blockchain, public and private. Other variations are hybrid and consortium.  Table 1 illustrates their purpose and some real world examples.

### 2.3. Blockchain Algorithm

The mechanism involving addition of chain of records and there after validating transactions is referenced as a blockchain algorithm. In blockchain consensus algorithms, each new block added to the network is agreed by all the nodes in a distributed/decentralized computing network.  Table 2 lists some of the important blockchain algorithms since 1993.

### 2.4. Blockchain Algorithm

In the recent years, there have been several blockchain initiatives. Following are some of major domains where blockchain has provided a secured way of transferring the data between the various users.

- Financial: fast transfer of funds, smart contracts, equity trading, e.g., Blockchain.info [3]
- Product tracking and tracing: agriculture food supply chain, weapon tracking, logging the resources, e.g., Walmart Food Safety cooperation (with IBM and Tsinghua University) [4]
- Business: retail management, managing gift cards, and loyalty cards, e.g., BoardRoom [5]
- Legal: copyright and royalty, real estate, transfer of will, notary, and worker's right, e.g., Cadastres (ONG Bitland in Ghana)—Digital land registry project in Ghana [6]
- Medical: medical record keeping and tracking of drugs, e.g., Blockchain Health [7]
- Authentication of ID and digital voting, e.g., Follow My Vote—an open-source online voting software [8]
- Backup: intermediary repository of unused data of industries for further sharing and selling and backup of data centers, e.g.,: Storj [9]
- Entertainment, e.g.,: Mediachain Labs' purpose is to provide connectivity between artists and other right holders with the tracks hosted by Spotify services [10]
- Social, e.g., Matchpool—a blockchain-based matchmaking platform [11]
- Education, e.g., certificates through blockchain (Holberton School in San Francisco) [12]

## 3. Blockchain in Healthcare

The advent of blockchain technology in healthcare services can reduce the healthcare fraud. The inculcation of Blockchain technology can transform the whole healthcare paradigm by making it more patients centric. It encourages the secured communication of data between the different stakeholders in a secured environment. Figures 2–4 illustrate different stakeholders and their relation in a blockchain-based healthcare system.

The medical data is fragmented and is distributed across different departments and providers. As both the number of patients and complexity of their ailments are increasing rapidly, the quantum of data that the hospitals have to handle every day is growing rapidly. The data is of many types like patient health information, EHR, medical insurance claims, and even IoT devices generate a lot of data. The most crucial aspect in providing proper medical services is to completely secure the methods of information sharing. These allow healthcare providers and all other stakeholders to verify the correctness of data. This is where blockchain comes in use. Some of the advantages of incorporating blockchain in healthcare are as follows:

- Data integrity: this can be achieved by verifying the data timestamp and perform unchangeable medical audits. There is no need to rely on third-parties which will definitely reduce the audit cost and ensure data safety.
- Drug traceability: fraudulent drug dealers can be easily detected in a blockchain-enabled transactions as they are timestamped and immutable. Whenever the drug is manufactured and moved to the retailer, the operational data is recorded on the blockchain. The whole path of the drug movement can be easily verified and all the chain links can be accessed at any point of time
- Data security in clinical trials: the users can prove the authenticity of the clinical documents registered in the system through blockchain technology
- Patient data management: in a blockchain-enabled system a hash is created for each PHI (patient health information) block along with the patient ID. With the help of appropriate API, the entities can access relevant information without revealing the patients identity. Similarly, the patient can also decide to whom they give access and its level (full or partial).
- Improve medical record access and record keeping: the electronic health record (EHR) of a same patient may differ from one healthcare provider to another healthcare provider, so its maintenance is a challenge. The blockchain-enabled system shall allow the transfer of records from one doctor to another as per the requirement
- Cutting costs and time: the data in medical domain is distributed in various agencies. Accessing the medical history of the patient from the previous healthcare provider consumes time as well as money. Application of blockchain in healthcare services can reduce both. Besides, the physician's credentials can also be verified

Table 3 provides the list of some popular initiatives in the healthcare domain where blockchain has been applied and made the system more secure. In the recent years, there is a significant impact of blockchain in the medical domain.

### 3.1. Blockchain in Covid 19

Healthcare is one such domain that has been the worst-hit during the ongoing pandemic. The greatest challenge faced by most governments and international organizations was to create a precise mechanism that can examine the cases discovered of the ongoing pandemic and predict the risk of its spread. An innovative solution is needed to fight against the battle of COVID-19 emergency [22].

During this pandemic crisis, the upcoming technology of blockchain can play a significant role in medical healthcare by handling various data related to patient's record, vaccination report, and the supply chain of drugs from the producer to the patient.

The patients' health record can be handled more securely over its peer-to-peer network. Through blockchain technology, the previous ailments of patients facing the symptoms of Covid-19 can also be found in the records. The concerned government and local authorities can only view this secure data for monitoring and further action [23].

Vaccination has become an essential requirement during the COVID-19 pandemic by the government for all the citizens. Blockchain technology can be used to create a more safe and secure vaccination system. A data storage infrastructure can be made to connect the vaccination records. The system implements a blockchain that can restrict unauthorized access [24].

The inclusion of blockchain can improve the management of clinical data and can streamline the communication between diverse stakeholders of the supply chain etc. The pandemic has increased the spread of misinformation causing panic among the public and irrational behavior. The new blockchain tracking system can review and authenticate all the information received by the public and the government. A study by [25] reviews the opportunities that blockchain provides in combating the disease by developing a tracking system for the data collected of the COVID-19 patients from multiple sources. A blockchain system using Ethereum smart contracts and oracles is being implemented to track the new and recovered cases and total deaths. In addition, security analysis is also provided along with the incurred cost by the stakeholders and their future work direction.  Figure 5 depicts the various applications of Blockchain during COVID-19.

### 3.2. Supply Chain Flow for Vaccination Distribution

In the hospitals and pharmacies supply chain, there are many stages involved like packaging, manufacturing, distribution, and regulation of the drug at hospitals and pharmacies. During this flow, it is not easy to track and ensure authenticity at each stage. With blockchain, it could significantly improve supply chains, and it would be able to provide greater security.

In the distribution of COVID-19 vaccines, temperature has to be monitored and enough storage time is essential. Blockchain along with IoT sensors can be used for transportation, collection, and storage of vaccines. It can allow the hospitals, distributors, and regulators to have a track of vaccination along with their data. It will also help to check whether the vaccines are stored and transported correctly.  Figure 6 demonstrates the applications of blockchain during the various stages of vaccination distribution.

Blockchain technology can plays an essential role in the battle against the ongoing pandemic. Many applications were developed. However, most of them are not mature enough to reveal their expected impact. Further studies are required and still going on in this area.

### 3.3. Blockchain in Indian Healthcare

In India, the inclusion of blockchain is growing gradually. In the year 2013, the RBI has taken cognizance of the fact that cryptocurrency is being used widely in open markets across the world. It has cautioned users, holders, and traders towards using “Virtual Currency” for any purpose but it remained silent about legality of its use [26]. Responding to the RBI views, most of the exchanges dealing in cryptocurrency scaled down their operations from 2017. These operations took a further hit when RBI, in April 2018, banned all banks and financial institutions under it, from either dealing directly or providing any service to any entity dealing with cryptocurrency [27] but recently, the Reserve Bank of India (**RBI**) has lifted ban on crypto exchanges.

There are seven key stakeholders in Indian Healthcare ecosystem—patient, provider, payer, pharma, medical technology, technology vendors/suppliers, and the government/healthcare regulator. The level of protection is dependent on the type of communication. Different solutions have been proposed in this regard. The authors of [1] have designed communication layers in Indian ehealth system according to the level of sensitivity. Indian ehealth system makes use of passwords, smart cards, etc. Although the usage of blockchain in healthcare services is in its infancy and India is pacing towards its adoption and inclusion. Indian government has recently started working on a national framework aimed at supporting wider deployment of blockchain use cases like land records (creation of a new blockchain enabled system for managing land record transfer and ownership), pharmaceutical drug supply chain, SuperCert (blockchain solution for educational certificates), immunization supply chain, insurance, and organic farming [28, 29].

Table 4 specifies some of the Indian blockchain initiatives in the field of health services.

Besides this, according to [30] CallHealth, which is considered to be world's first fully integrated healthcare platform dealing with all aspects of health, in partnership with ThynkBlynk, is trying to start India's first cross industry undisputable data-interchange using blockchain. It has the capability to integrate data with full security from all types of healthcare services and healthcare ecosystem providers like doctors, nurses, hospitals, clinics etc., while being fully compliant to stringent data privacy regulations and will address various issues like verification of fake and fraudulent data and the cost involved in repeated clinical trials shall also be reduced [31].

## 4. Literature Review

The following section provides a brief literature review about the role of blockchain in the domain of healthcare. The publications have been taken from IEEE explore and Science Direct. However, in 2008, with the introduction of “Bitcoin” which is a cryptocurrency, blockchain gained popularity but utilization of blockchain in healthcare started picking up since 2016. The methodology for collection of publications is shown in Figure 7.

MedRec is a system for handling EMR (electronic medical record) using blockchain technology which has been proposed by the authors of [32]. This system facilitates the users to access their medical information securely with much ease. Two protocols were designed in [33] for healthcare based on pervasive social network. The first protocol that displays authenticated association is an improved version of the IEEE 802.15.6 and second protocol shares health data among various PSN nodes using blockchain technique. The report [34] aims to illustrate possible influences, goals, and potentials connected to this disruptive technology. To understand this concept and its applications better [35], aimed at reviewing the available information on Healthcoin.

The paper [36] illustrates measures to evaluate DApps based on blockchain in terms of their compliance, feasibility, and intended capability in the healthcare domain. The motivation behind the study [37]is to devise client driven well-being information sharing arrangement by using a decentralized and permissioned blockchain and upgrade the character the executives utilizing the participation administration. The paper [38] investigates current procedures and plans to present a defense for blockchain innovation as an improved security model that can possibly bring down the expense of trust and an option in contrast to dealing with the weight of confirmation.

In [39] the creators have introduced and exhibited the utilization of blockchain innovation in numerous mechanical applications. The foundation of HealthChain, which is a healthcare industry application in blockchain, formulated and developed using IBM blockchain initiative. The authors in [40] tried to investigate different blockchain structures, analyzing existing challenges, and provide possible solutions. The authors in this paper [41] design an efficient recovery scheme and lightweight backup for keys of health blockchain using body sensor network according to the features of health blockchain. A disruptive technology based on blockchain is implemented [42] which facilitates cryptographic security and data access for medical communities in a formalized way via smart contracts for the purpose of data security and to make this data accessible to doctor and other trusted parties.

In paper [43], a Blockchain-Internet of Things model to solve issues is proposed. In this model, real time data of a patient's medical status is measured and collected via a bio-sensor and is stored in the blockchain. The paper [44] portrays a blockchain design as another framework answer for flexibly. A dependable instrument for secure and effective clinical record trades has been proposed. To meet the overgrowing healthcare services demand, the Advanced Blockchain (ABC) approach was designed. In the paper [45], a parallel healthcare systems (PHSs) framework has been proposed with the objective of improving the accuracy of diagnosis and the effectiveness of treatment, this framework is based on parallel execution (ACP) approach, artificial systems, and computational experiments. With the integration of healthcare and smart cities [46], utilizing information and technology for healthcare and medical practices around the globe is possible now. With Blockchain technology only, it is secure and safe to store information of a patient in the health care system. The authors depict the harmonious connection between blockchain and smart cities in the article [47].

The paper [48] aims at simulating the time response of healthcare blockchain network based on PBFT (practical Byzantine fault tolerance) using continuous-time Markov chain (CTMC) models. The paper [49] concentrates on the study to build up a model of medicinal services administration application in dental facility administration. It has an exchange ID number that is produced by hash number component running by Hyperledger Composer. The paper [50] discusses about how to deploy blockchain technology in healthcare, evaluation of such deployments in this area, and hence reviewing the pros and cons of such an approach. A medical questionnaire management system based on blockchain for sharing information has been proposed by the authors of [51]. The paper [52] investigates the possible uses of blockchain innovation in current social insurance frameworks and features the most significant necessities to satisfy the need of such frameworks, for example, trustless and transparent medicinal services frameworks. A coupled AI-Blockchain EHR management system has been proposed by the authors of [53] for providing a platform that incorporates artificial intelligence (AI) and blockchain for the following: (i) secure EHR management, (ii) efficient data integration, and (iii) reliable computer-aided diagnoses. To support the decentralized healthcare cycle, the underlying technology required can be provided by smart contracts and blockchain by maintaining medical record integrity and patient trustworthiness.

Alexaki et al. [54] present a conceptual mechanism for sharing and accessing medical records. Such a mechanism is suitable for a system operating with healthcare judiciary regulations. The authors present CORUS, a system for evaluating healthcare remedy which uses crowdsourcing based on blockchain on a cloud computing platform [55]. CORUS is the premier system to leverage crowdsourcing, cloud computing, and blockchain for evaluating healthcare remedy. In the paper [56], the authors study the possibility to utilize the blockchain innovation to ensure healthcare services information hosted inside the cloud. The research proposal in [57] is about an accessibility mechanism in a given healthcare system for the patient and the doctor in an efficient and secure manner based on blockchain. The authors have proposed a blockchain-based smart contracts to manage medical devices and information of patients with the objective to protect information that is private and device-generated [58]. In paper [59], the authors have provided solutions for utilizing personal health data in healthcare which is blockchain enabled and also discusses issues and challenges associated with it.

Theodouli et al. [60] present the capability of blockchain technology to ensure the following: (i) private and auditable healthcare data sharing and (ii) healthcare data access authorization handling by proposing a system architecture design based on blockchain. There is a two-fold requirement to prevent impermissible accessing of health data of patients as well as making such data easily accessible to patients [61]. One possible solution may be blockchain. The authors of [62] have proposed a blockchain-based framework for efficient storage and upkeeping of EHRs which ensures reliability and efficient healthcare data accessibility by patients, providers, and third parties, while taking care of the patient's privacy. BlocHIE is a blockchain-based platform for healthcare related data transactions [63]. The paper [64] presents a framework that utilizes a blockchain and an off-tie brought together information stockpiling to give patients and clinical experts moment access to their clinical records from anyplace. It is now believed by many experts that leveraging blockchain technology [65] might be beneficial to get a patient's appropriate medical information from where it is stored to where it is required, as well as allowing patients to view their own medical histories easily

In this work [66], the authors have proposed a new blockchain-based model that ensures the GDPR compliance. This is accomplished by handling references to the sensitive data and instead of manipulating private data directly, metadata is used within the blockchain. In [67], a proposal has been made for BBACS (Block-based Access Control Scheme) that provides an access control solution for transacting electronic medical records (EMRs) which is blockchain-based. BBACS contains an access scheme and model. The paper [68] presents a blockchain based innovation system for identification and access management that can be used as a backend in a digital system to provide authorization and authentication. The paper [69] focuses on leveraging blockchain for smart homes and healthcare with the objective of improved privacy and security. The paper [70] proposes a signature scheme for healthcare based on blockchain. It is decentralized and attribute-based, which provides efficient authenticity verification of EHR data and signer's identity taking care of privacy. In [71], the authors have presented conceptual design for sending personal healthcare information which is continuous and dynamic in nature using blockchain technology supported by cloud storage secured with transparency. The study proposed in [72] is about a centralized, secure, and authenticated blockchain-based system for healthcare in developing countries using Hyperledger.

Paper [73] presents an IoT and blockchain-based platform architecture to facilitate the diabetes treatment and assist patients for its proper self-management. The authors in [74] have proposed BPDs based on blockchain for the purpose of maintaining privacy during data transaction for EMRs. In BPDS, the indexes are reserved in a tamper-proof consortium blockchain and the primitive EMRs are stored in the cloud securely. The objective of paper [75] is to design a diagrammatic and conceptual medical app model that is capable of maintaining a complete patients' and doctors' database in case of a surgery using blockchain technology. In the paper [76], the authors have presented a framework called “EMRShare” organized in a cross fashion based on authentic blockchain innovation to provide solution for reliability issues prevalent in EMRs transaction activities. The paper [77] proposes GAA-FQ (Granular Access Authorisation supporting Flexible Queries) as architecture for blockchain-based electronic medical records (EMRs) comprising of a model and an authorization scheme for accessibility.

Paper [78] gives an overview of the major concerns associated with the analysis and security of healthcare information thus providing the solution for improved healthcare services. In accordance with the health blockchain features, the authors of [79] design a scheme for backup and recovery scheme that is lightweight and efficient, respectively, by using a body sensor network for keys of health blockchain. The paper [80] tries to utilize blockchain technology for improving the security and interoperability of EMR systems. This in turn will benefit various participants in health sector of countries like Kenya. Paper [81] explores an attribute-based signature scheme with multiple authorities. This ensures validation of EHRs encapsulated in blockchain, in which a message is endorsed by a patient as per the attribute while disclosing no information except the evidence attested by himself/herself. The research done by [82] is aimed at identifying a conceptual blockchain-based eprescription system. The system leverages the principles of cryptocurrency for its application in eprescription processes to accomplish the goals.

The authors of [83] emphasize on safe data storage and transmission using lockers as an effective measure. The strengths and prospects of implementing blockchain for managing socioeconomic systems are also presented. Work is as of now in progress to bring blockchain innovation to the medicinal services industry [84], and administrators of hospitals are trying to envisage its use for clinicians, patients, and for themselves. It also involves chairmen at Beth Israel Deaconess Medical Center, which is mainly a scholarly medical institution located in Boston, USA. The article [85] tries to present an attribute based scheme meant for control of access as an addition with controlled access delegation capabilities which can work in a multidomain ehealth environment. The paper [86] proposes an access control manager which allows access and storage of data in a secure manner. This is further utilized by the classifier while doing real-time retraining via external data storage location. A Proof of Disease (PoD) consensus protocol, which has a basis in Ethereum alongside a single instance of truth which can be understood by the computer, is discussed in the paper [87].

The paper [88] has a new method, process, and system to calculate dyslexic symptoms to generate a metric data. This can be generally used by any individual, community, or a group. Paper [89] presents an in-home therapy management framework that provides support for low-latency, anonymous, secure, and continuously accessible spatiotemporal multimedia therapeutic information interaction within an on-demand information-sharing scenario by utilizing the IoT nodes and the blockchain-based decentralized MEC. Building on existing blockchain technologies, researchers [90] from both academic and industrial sectors are exploring applications including fraud detection, identity verification, and smart contracts that are concerned with use in healthcare. Discussion in chapter [91] revolves around the current healthcare data security concerns as well as existing and futuristic regulations on this sector. Blockchains can deliver these transactions in a transformative manner by using smart contracts as a catalyst in healthcare [92]. By utilizing the distributed [93] or decentralized property, blockchain innovation guarantees the responsibility and integrity. Various solutions have also been provided using decentralized methodology to control the impact of attacks.

In [94], the mind boggling nature of acts performed by people in different healthcare environmental conditions lessens the subjective measures for extricating particular highlights speaking to different human activities. A framework based on multiclass cooperative categorization strategy to keep a check and acknowledging such activities, which depends on multiclass helpful order strategy has been proposed in response to this challenge. In paper [95], the authors have worked for searchable encryption scheme for EHRs using blockchain. The indexing for EHRs stored in the blockchain is done using complex logic expressions. In [96], for patients and health professionals, the personal health record (PHR) and electronic health record (EHR) play a prominent role in efficiently accessing health records data. However, an integrated visualization of health data that is distributed across different health providers is difficult to obtain.

The main objective of the study [97] is to propose a new verification framework which is secured for verifying authenticity of a patient between an access point and a node database. Blockchain initiatives such as MedRec, voice assisted interfaces, such as Alexa, Siri, Google Now, and chatbots viz. Woebot are among the emerging technologies in the area of mobile health [98]. The qualities and shortcomings of these advanced digital tools have also been discussed in this chapter. The paper [99] aims at implementing B2B/G2B-based electronic payment along with General Ledger auto-reconciliation system via a highly complex project which demands powerful and advanced cyber-security technologies. The paper [100] is concerned with smart healthcare sector to maintain the privacy of patients' data as well as providing medical practitioners with reliable and real time accurate data. In [101], the stress of noncentralized database in blockchain technology is on data sharing. The blockchain technology consensus ensures legitimacy and security of data.

The paper [102] has contributed in the following ways: (i) results reporting of a systematic literature review; (ii) summarizing and categorizing existing benefits/challenges on leveraging blockchain in healthcare domain; (iii) providing a framework that will promote innovative research activities; and (iv) establishing the evidence state with deep assessment. In the paper [103], the authors focus on implementing the key aspects of blockchain to a health application network where health related data of patients can be leveraged to alert authenticated and verified healthcare providers about important information with security and privacy. In paper [104], DASS-CARE, a framework based on blockchain for easily accessing healthcare services and medical records in a scalable, secure, and decentralized manner has been proposed. The proposal in [105] is to keep encrypted EMRs in the blockchain, and the decryption key is shared by a patient only with trustworthy healthcare professionals. The paper [106] guarantees total security, integration, and access control of appropriate ehealth records to the data proprietors during its conveyance on the blockchain.

The paper [107] addresses interoperability concerns: disparate systems and medical data in silos. The paper [108] highlights the usage of Internet of Things (IoT) and blockchain in the healthcare domain, recognizing the scope of using these new digital technologies to enhance current methodologies. In the paper [109], authors try to explore blockchain-based technology to facilitate healthcare data handling with respect to cybersecurity, regulatory frameworks, patient rights, and provider-centric perspectives. Paper [110], discusses the dual nature of blockchain model for the healthcare domain. The model unifies private patient blockchain and healthcare authority blockchain for building a tamperproof permission tracking system to guarantee increase in security and privacy while improving redundancy in permission and record. In the paper [111], presents a scheme called as ABE for achieving the dynamic authorization and authentication for the MoD services in telemedicine system in an efficient and flexible manner. During alteration in an ordered service by a patient, the following issues needs to be dealt with privacy of data; cryptography; data security; Internet; Internet of Things; computer network security; authorization; contracts; cryptocurrencies; and cloud computing [112].

In the paper [113] authors have proposed a novel framework on a mobile cloud platform by combining decentralized interplanetary file system (IPFS) and blockchain for sharing EHRs. HealthChain [114] is a scheme for maintaining privacy of healthcare data based on blockchain on a large-scale, by encrypting health data for conducting fine-grained access control. The application of HealthChain for smart healthcare system is very well shown by experimental results and security analysis. The paper [115] portrays blockchain as a distributed transactional system of record that can provide underpinnings to enable these transformative opportunities and trends HCLS by providing secure and authenticated transactions, immutable data on a shared ledger, and smart contracts that can represent rules that are executed with secure transactions. In the paper [116], the main motive is to do a performance-based investigation of trust management based on blockchain with focus on a specific type of IoMT named as medical smartphone networks (MSNs). The paper [117] discusses a proposal for a blockchain-enabled authorization framework for management of medical files and IoMT devices both by creation of a distributed custody chain and health data privacy scheme.

As per discussion in [118], combining blockchain with the Internet of Things (IoT) and then applying it as a catalyst will process these transactions to disrupt healthcare from its current state at this time. In the paper [119], architecture for applications in ehealth based on blockchain has been proposed. It provides for a confidential access control mechanism efficiently. It utilizes key features of blockchain during modification of the classic structure of blockchain like anonymity and immutability users in order to overcome its challenges faced in IoT applications.

The paper [120] focuses on incorporating blockchain technology for securing remote patient monitoring-based systems of Internet of Things (IoT). The paper presents the advantages and furthermore functional impediments of blockchain-based security approaches in monitoring patients remotely by utilizing IoT devices. The workstream prestandards [121] made way for developing IEEE SA Standards efforts recommendations for making Clinical IoT data and device interoperable with mnemonics as TIPPSS-Trust, identity, privacy, protection, safety, and security-in connected healthcare to improvise outcomes of healthcare and data sharing. In the paper [122], different methodologies for healthcare concerns are discussed by various researchers in the area of IoT. A theoretical analysis of proposed solution is performed at the end. A detailed review of the present blockchain customs has been introduced for the Internet of Things (IoT) structures [123]. It is able to change way of life of numerous people in a few zones effectively because of its extreme effects on organizations and ventures despite a lot of questions regarding its adaptability, supportability, and security by commentators..

The authors of [124] have done a comparative analysis of core blockchain architecture, along with fundamental concepts, and its applications in three major areas: business and automobile industry, healthcare, and the Internet of Things (IoT). The work in [125] presented is based on an blockchain-enabled IoT system that improvises challenges faced in storing data of patients received by wearable IoT devices thereby helping medical practitioners to make decisions that are much informed on the basis of efficient medical record-maintenance.

In the paper [126], a scheme for monitoring outdoor health securely in a smart city is proposed that is based on blockchain and uses UAV (Unmanned Ariel Vehicle). The scheme proposed is concerned with accumulating health data from inbuilt sensors in wearable of users and transmitting this data to the MEC server which is nearby through UAV. The paper [127] analyses the users and state-of-the-art expert's views to explore the societal and technical barriers involved in SHS adoption. One SHS framework to provide intrinsic system security and integrity based on blockchain has been proposed further. The future exploration bearings and use instances of blockchain in healthcare area are also talked about in final terms.

In the paper [128], authors have proposed a completely new protocol named as Pseudonym Based Encryption with Different Authorities (PBE-DA) for achieving perfect confidentiality maintenance for patients in order to meet the requisites of distributed structure in the ehealth records (EHRs) system. This is accomplished by the application of blockchain concepts on the entities of healthcare communication in an electric health platform. The paper [129] deals with analyzing blockchain-IOT impact in the healthcare industrial sector. The article [130] does a comparison between the traditional EHR systems using client-server architecture and the blockchain enabled systems. The authors of paper [131] propose a secure healthcare scheme using a blockchain technology where health data is collected from users using unmanned aerial vehicle (UAV). The data is then stored in the nearest server [132], discusses the blockchain applications in the radiology field. The paper [133] discusses the role of authenticated and permissionless blockchain and its potential implementations. The chapter [134] gives a stress on the use cases of healthcare and blockchain applications, along with the technical challenges faced, that are being addressed by blockchain developers and researchers in recent times worldwide.

The survey [135] results have shown the distinct advantages of blockchain for healthcare applications in comparison to other applications. The work done in [136] portrays a holistic view of applications and fundamentals of blockchain for healthcare and thus helping to plan and strategize the blockchain-based technology usage. The study [137] gives a systematic review, assesses, and synthesizes publications that are peer-reviewed for leveraging/proposing to leverage blockchain for improving healthcare services and processes, health education, and health sciences.

The paper [138] talks about the different challenges faced in the healthcare security and exploring its solution via blockchain technology. GuardHealth is an effective, reliable and distributed blockchain system for exchanging data and maintaining data privacy [139]. The study [140] explains the current status of work in applying blockchain in healthcare sector with discussion on the contributions made by customized blockchain models of four-layers that is connected to precision medications and clinical trials. A decentralized off-chain medical data repository [141] that uses IPFS (InterPlanetary File System) and blockchain technology has been proposed that might maintain patient's privacy. The article gives a review [142] for the purpose of identifying how blockchain addresses extensibility issues and solves the issues in the healthcare domain by implementing blockchain innovations. An EHR auditable trail access and a procedure for transparent insurance claim for healthcare providers using smart contracts have been introduced in [143].

The paper [144] proposes a PHR on the basis of Hyperledger Fabric (consortium blockchain). It further analyses and compares the performance on the basis of delay in transaction and ledger size.

The creators of [145] have proposed a new decentralized confirmation of patients in a distributed emergency clinic arrange, by utilizing blockchain. In article [146], a data-flow architecture to combine IoT and blockchain called as IoBHealth has been proposed. It can be used for accessing, managing, and storing electronic healthcare data. The architecture proposed in [147] based on blockchain has been designed and discussed for exchanging personal health report (PHR) of a patient among the different health organization parties in a secure manner with ease. In [148], computer scientists, healthcare/IT professionals, and healthcare providers as well as medical researchers come together with the objective to raise the availability of SDI (software defined infrastructures) while fulfilling the performance and regulation requirements of applications of healthcare with the help of blockchain.

The paper [149] is about BioMED, a Blockchain-based framework to improvise data integration and interoperability with concern to EHR-sharing. The solutions proposed inculcates an access management system that permits exchanging EHRs between a distributed trusted third party auditor (TTPA) and different medical providers that ensures data integration. A DIT IoHT utilizes a private blockchain ripple chain and is devised for establishing reliable data exchange by nodes validation. It is based on the interoperable structure to enable controlled communication necessary for solving issues related to fusion and integration being available through different zones of the IoHT infrastructure [150]. The motive of paper [151] is to investigate the verification impact on trust level among the distinct health data-trading system entities by an evolutionary game theoretic model proposal. The paper [152] motivates the investigation of using blockchain technology for managing identity and data of a patient. A few promising issues and directive research on blockchain-helped secure EHRs in cloud-based ehealth frameworks have been examined in [153]. The paper [154] tries to study and provide solutions for universal storage of health records in recent healthcare analytics and solving the problem of collecting personal health data generated via wearable devices. The paper [155] portrays an extensible architecture for exchanging digital health records via a Hyperledger blockchain which is multi-channel. The article in [156] is about proposing a new Bitcoin-IoT node-based lightweight system model while integrating the improvised and simplified payment verification (SPV) method for e-healthcare application. The paper [157] explores the novel pharmaceutical administration dependent on IoT and Blockchain innovation.

The authors of [158] have thrown light on the blockchain process of providing certificate for the health services. In [159], a structure has been devised combining blockchain with edge computing for leveraging security, scalability, and privacy to the medical domain. The use cases also play an important part in deciding the new norms for security. In this regard, the article [160] illustrates some use cases leveraging the solutions based on blockchain which shall helpful in organizing the medical records. An authentication protocol for the IoT-enabled medical system BAKMP-IoMT has been designed in [161] for maintaining the security issues between implantable medical devices, personal servers, and the cloud servers. Security of medical records is one of the pertinent things in healthcare services. The authors of [162] have analyzed the usage of blockchain technology in providing security and storage of medical records for United States health services from industry perspective. In [163], the application of different technologies like blockchain, artificial intelligence, 5G, unmanned ariel have been discussed for combatting the pandemic COVID-19 outbreak. The authors of [164] have thrown light on the design and development of the model based on blockchain for imparting security and privacy of data and ensuring that the patients get full control of their health records.

## 5. Analysis

This section provides the analysis of the literature review provided in the previous section. The total number of publications in conferences, Journals and symposium/workshops has been shown in Figure 8.

It can be observed that maximum number of publications is through conferences.  Table 5 shows the number of publications of blockchain in healthcare since 2016. It can be analyzed that the usage of blockchain has been increasing constantly. The corresponding graph of this table has been shown in Figure 9.

Further a categorization has been done to illustrate usage of blockchain in the different healthcare sectors. The different categories defined here are challenges and benefits, access management, EHR, evaluation and analysis, storage of data, and IOT/AI with blockchain.

It can be seen that maximum publications are in the category of IOT/AI with blockchain. The same has been mentioned in Table 6, Figure 10, and Table 7.

Total 148 papers have been reviewed, and maximum number of studies is in the area of analyzing the various challenges and benefits by involving blockchain in healthcare followed by blockchain enabled services with IOT. It can be observed from the Figure 11 and Figure 12 that there is a constant rise in these domains.  Figure 13 provides information about the year wise publications in the different categories in the five consecutive years 2016, 2017, 2018, 2019, and 2020. The specific details in the year 2018 and 2019 have been presented in Figures 14 and 15. It can be observed that maximum publication is in the area of EHR in 2018 and in the category challenges and benefits in the year 2019.

## 6. Issues in Blockchain Technology: Disadvantages and Challenges

The advantages of blockchain in healthcare are plentiful and have the ability to transform the entire sector. There are certain issues which are causing hindrances in its wide deployment. Mass adoption is required for the improvement in the entire healthcare system. List in Table 8 are some major disadvantages and challenges in the global acceptance of this technology.

## 7. How This Study Is Different from the Previous Study

The study has provided the review of 148 publications focusing on the integration of blockchain technology in healthcare. Following are the major unique focus areas:

(i) The manuscript discusses the role of blockchain during COVID-19
(ii) The paper throws light on the prospects of blockchain in Indian scenario
(iii) It consolidates the various issues related to blockchain like algorithms used, details of companies who have taken initiatives in incorporating blockchain in different applications
(iv) Categorization of publications on the basis of conferences, journals, and symposium/workshops
(v) The number of publications as per chronological order (since 2016).
(vi) Publications have been categorized and analyzed on the basis of following heads:-
  1. Challenges and benefits
  2. Access management
  3. EHR
  4. Evaluation and analysis
  5. Storage of data
  6. IOT with blockchain
  7. Protocol/algorithm
  8. Model/design
  9. Disease/diagnosis
  10. Others (integration with AI and Cloud, SHS, smart cities, smart contracts, and UAV)

## 8. Recent Studies in Blockchain Technology

This section describes some of the recent publications on the applications of blockchain technology in the healthcare domain.  Table 9 throws light on some of the recent publication in this domain.

## 9. Suggestions

Postarrival of Industry 4.0, all fields of work have deployed or are in process of deploying solutions based on cutting edge technologies like artificial intelligence, machine learning, IoT, and blockchain. Healthcare is certainly no exception. No doubt the wide deployment of blockchain-enabled healthcare system will definitely revolutionize our lives. Improvements are still required for seamless blockchain adoption across medical industry.

- Blockchain with Data Analytics and AI—the inclusion of AI in blockchain enabled healthcare system can increase the efficiency of medical staff and democratize healthcare. It can make the data more coherent, and understandable, and determine the logic which shall be helpful in decision making process. The application of AI can also fill the gap of staff shortages in healthcare. By using predictive and descriptive algorithms, ML is fundamentally improving usage of existing data for identification of patterns and forming new insights. The combination of the two technologies mention above will surely speedup data exploration and analysis while at the same time enhancing transactions security.  Figure 16. depicts the function of blockchain and AI as used in the medical domain. It depicts as to how structured and unstructured data flows through various components of healthcare system. It further shows how meaningful insights can be derived from the available as well as collected data by using artificial intelligence and blockchain technology
- Easy to use Blockchain Tools and Platforms—the initial establishment of blockchain infrastructure costs is high and for making this technology effective and adaptive, it is pertinent to focus on that solution which can help in easy deployment and thereby reducing the cost. In this regard, cloud services can be utilized by offering blockchain as a service to the users. This will surely result in the reduction of cost and complexity. Blockchain networks can be run on the specified templates reducing the barriers of operating blockchain network
- Big Data Blockchain—the amount of data generated in healthcare industry is enormous and carries diverse variety. The data is in both structured and unstructured formats. Blockchain-based big data platform can enable large and complex data specifically designed to support global interoperability which can bring data from various sources. The main advantage is that it can significantly broaden medical knowledge and reduce operational costs. The different kinds of medical records like patient history, treatment plans, imaging, insurance information, etc. can be simplified by drawing a pattern from it. This pattern later can be shared among clinicians and medical research companies for diagnosis and treatment
- Awareness and Skill Development—the wide deployment of blockchain technology in any organization demands its awareness as well as upgradation in the skills of the employees. Special awareness programs and training/workshops should be conducted to make the system blockchain enabled

## 10. Conclusion

In today's industry, data has become one of the most crucial aspects. Its importance cannot be emphasized enough in the healthcare sector. The management of huge data in healthcare is costly and error-prone and therefore challenging. With the advent of blockchain technology, the medical domain can have a trusted and secured system. This technology has the potential to completely transform the delivery of care by the healthcare industry and specially, how an individual can access care, anywhere in the world.

The study emphasizes on the importance of blockchain in the health domain. Some key outputs of the present study can be marked down as following:

- Blockchain technology has undoubtedly provided the world with an innovative disruption across a wide range of health services, but at the same time it has its own challenges which contribute to the lack of mass adoption. Few steps have to be executed to eliminate these challenges, and keep the momentum of blockchain adoption pointing upwards
- In terms of Indian scenario, it can be observed that there is a gradual growth for implementation of blockchain technology in healthcare domain. This is quite understandable for a developing country like India due to the energy consumption and cost involved in setting up of infrastructure
- Literature clearly reveals that in order to establish the competence and authenticity of blockchain technology, researchers are paying a lot of attention to the challenges and benefits associated with blockchain technology. The authors were able to shortlist as many as 14 articles in the domain of challenges and benefits for the year 2020 which is significantly more than the articles published in other areas. Total number of publications in this domain are 36
- IoHT is another area which has clearly attracted the researchers with as many as 27 publications since 2016 and 19 publications in the year 2019. This indicates the visualization of researchers for combining IoHT with blockchain to have a powerful impact on managing different aspects of healthcare domain
- Leveraging the potential of technologies like artificial intelligence, machine learning, data analytics, and big data into blockchain have also become an area of interest for the researchers to empower the health services
- Out of the seven categories selected for review, very little work has been done on ‘storage of data', which is a crucial aspect of blockchain and more research is required in it
- Researchers also analysed the impact of blockchain during a pandemic as that of COVID-19 and suggested various domains like tracking of the production of vaccines, checking their quality etc.

Blockchain is a powerful technology that can bring a significant change in the healthcare domain. However, lot of research and investigations are still needed to make this technology acceptable to the masses. Through this paper, we have tried to bring forward the research and development in the area of blockchain technology. We have tried to include most of the relevant papers in this study but in case we missed an important article, we apologize for it.

## Figures and Tables

**Figure 1:** Advantages of Blockchain.

**Figure 2:** Process of Blockchain.

**Figure 3:** Blockchain in Healthcare.

**Figure 4:** Stakeholders in Healthcare.

**Figure 5:** Applications of Blockchain in COVID-19.

**Figure 6:** Blockchain in supply chain for vaccination distribution.

**Figure 7:** Methodology of search.

**Figure 8:** Publications in conference, Journals and symposium.

**Figure 9:** No. of publications since 2016.

**Figure 10:** Categorization of publications.

**Figure 11:** Challenges and Benefits.

**Figure 12:** IOT with Blockchain.

**Figure 13:** Year wise publications.

**Figure 14:** Year 2018.

**Figure 15:** Year 2019.

**Figure 16:** AI with Blockchain.

**Table 1:** Types of blockchain.

S.no.	Type of Blockchain	Purpose	Example
1.	Public	Non-restrictive, permission-less distributed ledger system.	Bitcoin, Litecoin, Ethereum
2.	Private	Operating in closed network as restricted or permission based blockchain.	Multichain and Hyperledger projects, corda.
3.	Consortium	Semi-decentralized type, greater than one administrator or organization has management rights to blockchain network	Energy web Foundation, R3
4.	Hybrid	Mixture of the public and private blockchain network. Using combination of feature of both types of blockchains enabling a private permission-based system and public permission-less system	Dragonchain.

**Table 2:** Blockchain algorithms.

S.no	Name of the algorithm	Year	Invented by	Purpose
1	Proof of work (PoW)	1993	Cynthia Dwork and Moni Naor	Creates new blocks in sequence of chain and also confirm transactions occur in each block.
2	Proof of stake (PoS)	2011	Sunny king	All blocks of chain are validated on the basis of strut of participants of network.
3	Delegated proof-of-stake (DPoS)	2014	Daniel Larimer	It works like voting system so participants vote to help the state of new block according to validators.
4	Proof of burn	2014	Lain Stewart	Works to reduce rate of energy consumption.
5	Proof of elapsed time (PoET)	2016	Intel	All participants of networks will wait for randomly time period, then who finished on time get new block and validates that block.
6	Proof of space	2015	Dziembowski.	Usage of space instead of computation is predominant in this algorithm rest of the functionality is very same as to proof of work algorithm.
7	Delayed proof of work (dPoW)	2016	Komodo project	It is a security mechanism that make use of bitcoin blockchain hashpower to enhance network security.
8	Proof of authority (PoA)	2017	Gavin wood	It delivers comparatively fast transactions through a consensus mechanism.
9	Leased proof-of-stake	2017	A variant of proof of stake	Any participant has a possibility to lease out their balance to mining nodes and these mining nodes share a profit with participants.
10	Proof of weight	2017	MIT computer Sc. & AI lab	It is a mechanism that gives users a ‘weight' based on how much cryptocurrency they are holding.

**Table 3:** Blockchain in healthcare.

S. no.	Name of company/organization	Purpose	Year of launch
1.	Medical chain	This is considered as the first healthcare company which made use of blockchain technology for storage and utilization of [13].	2016
2.	Medrec	Its purpose is to save time, money, and duplication of procedures between various stakeholders of health system with the help of blockchain [14].	2016
3.	Nano vision	Integrating AI with blockchain to collect molecular level data on Nano tokens was the purpose of Nano vision [15].	2018
4.	Gem	It aimed at giving authority to patients over their medical records and genomic data through blockchain technology [16].	2016
5.	Simply vital health	The purpose is to empower the providers and patients to access, share, and move their healthcare data with the help of blockchain technology [17].	2017
6.	Tierion	Data storage and verification of data is done through this blockchain based startup [18].	2015
7.	Guardtime	Security of patient healthcare data is achieved through this system based on blockchain technology [19].	2008
8.	Cyph	The main aim is to ensure a protected communication and secure digital identities between different stakeholders of healthcare system [20].	2017
9.	Blockchain health	A blockchain-based system for medical research management [7].	2016
10.	Hashed health	Tries to increase transparency and accessibility of the credentials in health sector. Using professional credentials exchange, the verification of credentials and track record of all health professionals can be done by any member of the chain [21].	2016

**Table 4:** Recent blockchain initiatives in healthcare.

S. no.	Name of the project	Location	Key domains	Web link
1.	PSI PHI Blockchain labs	Faridabad	Supply chain, telecom, and healthcare	https://angel.co/company/psi-phi-labs
2.	Darwin labs	Gurugram	Healthcare, banking, trade finance, and insurance	https://www.darwin-labs.com/
3.	KrypC	Bangalore	Healthcare, financial services, and legal travel	https://krypc.com/

**Table 5:** Number of publications since 2016.

S. no.	Year	No. of publications	References
1.	2016	3	[32–34]
2.	2017	10	[35–44]
3.	2018	48	[45–89, 128]
4.	2019	46	[90–127]
5.	2020	41	[129–165]

**Table 6:** Categorization of publications.

Categories	No. of publications	References
Challenges & benefits	36	[22, 34, 39, 40, 46, 52, 59, 60, 78, 84, 90–94, 101–103, 107, 109, 110, 115, 124, 133, 135–138, 140, 142, 149, 152, 156, 160, 165]
Access management	15	[42, 57, 61, 63, 64, 66–68, 77, 85, 86, 106, 114, 155]
EHR	21	[25, 32, 53, 54, 58, 65, 70, 72, 74, 76, 80–82, 95, 96, 105, 113, 130, 144, 157, 159]
Evaluation & analysis	11	[35, 36, 38, 50, 51, 55, 94, 133, 148, 151, 163]
Storage of data	2	[62, 83]
IOT with blockchain	27	[22, 43, 73, 89, 100, 108, 112, 116, 123–125, 129, 130, 147, 153, 154, 162]
Protocol/algorithm	6	[33, 41, 48, 87, 98, 111]
Model/design	11	[37, 44, 45, 75, 79, 88, 97, 139, 141, 145, 161]
Disease/diagnosis	5	[49, 88, 132]
Other(AI, cloud, UAV, SHS, smart contracts, smart cities)	14	[23, 47, 56, 58, 69, 71, 99, 100, 126, 127, 131, 143, 150, 164]

**Table 7:** Year wise publications.

Categories	2016	2017	2018	2019	2020
Challenges & benefits	1	2	7	12	14
Access management	0	1	10	3	1
EHR	1	0	11	4	5
Evaluation & analysis	0	3	3	1	4
Storage of data	0	0	2	0	0
IOT with blockchain	0	1	3	15	7
Protocol/algorithm	1	1	1	2	0
Model/design	0	2	4	1	4
Disease/diagnosis	0	0	3	1	1
Other (AI, cloud, UAV, SHS, smart contracts, smart cities)	0	0	4	5	5

**Table 8:** Disadvantages and challenges.

Slow speed	Redundancy of data
Lack of awareness	High set up cost
Large energy consumption	Integration with existing system
Interoperability issues	Standardization issues
Authentication problem since no central authority	Regulatory issues

**Table 9:** Recent publications.

S. no.	Title of the paper	Brief description	Year
1	A blockchain-based electronic medical health records framework using smart contracts [166].	The purpose of the study was to implement infrastructure to access smart contracts.	2021
2	Semicentralized blockchain based distributed system for secure and private sharing of electronic health records [167].	The study throws light on the usage of decentralized systems data storage model in a centralized system for allowing data reproducibility. It also uses the blockchain for providing security to the patient's data.	**2021**
3	BlockHealth: blockchain-based secure and peer-to-peer health information sharing with data protection and right to be forgotten [168].	The BlockHealth solution ensures the secured communication of personal health data. The hash values of the data are being stored. The companies manage the health data in private databases which permits to delete data in compliance with the right to be forgotten.	**2021**
4	Framework to enable pharmacist access to health care data using blockchain technology and artificial intelligence [169]	The purpose is to integrate blockchain and AI for enabling the pharmacist to access to health data.	**2021**
5	Blockchain technology and universal health coverage: health data space in global migration [170]	The blockchain can empower in real time multiorganizational services and workflows among multiple users anywhere in the national healthcare systems around the world as it is anchored in the security, privacy, and medico-legal regulation of medical data. This is an innovative approach highlighting possible future directions in IT-supported health.	**2022**
6	Blockchain's coming to hospital to digitalize healthcare services: Designing a distributed electronic health record ecosystem [171]	The information processing theory (IPT) may enable design and validation of a blockchain-based EHR system. This can increase the storage of medical records and data exchange among healthcare providers. Few of the benefits in implementing a distributed network are improved quality, reduced medical errors in clinical domain, financial, and operational benefits.	**2022**
7	Blockchain-based governance models for COVID-19 digital health certificates: a legal, technical, ethical, and security requirements analysis [172]	The focus of this study is to analyze the requirements of a blockchain-based data governance model for COVID-19 digital health certificates. The authors discovered loss of the main advantages of blockchain in this model i.e., decentralization and anonymity.	**2022**
8	Is blockchain the solution to the challenges of reliable interoperability in the healthcare ecosystem? [173]	Health standards and smart contracts are some of the most challenging issues facing the interoperability of healthcare systems. This paper highlights issues for the interoperability of healthcare systems using blockchain technology. The authors try to identify a solution from a software engineering domain for this.	**2022**
9	Improved security blockchain for IoT-based healthcare monitoring system [174].	The authors aim to reduce required bandwidth and increase efficiency of data security and privacy. To this end, they use a technique called enhanced proof of work (E-PoW) consensus blockchain. This may be used for IoT-based healthcare monitoring system.	**2022**
10	Task offloading strategy with emergency handling and blockchain security in SDN-empowered and fog-assisted healthcare IoT [175].	The paper has a task offloading strategy with low-latency, centralized, reliable, and secure decision-making algorithm. It is also having a powerful emergency handling capacity (LSRDM-EH) and used in resource-constrained edge devices for task offloading. In order to provide security to the complete network, a blockchain-based, two-layer, multidimensional security strategy is mentioned.	**2022**
